The article "An Investigation of Regional Plantar Soft Tissue Hardness and Its Potential Correlation with Plantar Pressure Distribution in Healthy Adults" was published in 2021. Journal: Appl Bionics Biomech.

# An Investigation of Regional Plantar Soft Tissue Hardness and Its Potential Correlation with Plantar Pressure Distribution in Healthy Adults

**DOI:** 10.1155/2021/5566036

**Published:** 2021-06-12

**Authors:** Maimaitirexiati Helili, Xiang Geng, Xin Ma, Wenming Chen, Chao Zhang, Jiazhang Huang, Xu Wang

**Affiliations:** ^1^Department of Orthopedics, Huashan Hospital, Fudan University, China; ^2^Fudan University, China

## Abstract

**Background:**

The plantar soft tissue plays a critical role in absorbing shocks and attenuating excessive stresses during walking. Plantar soft tissue property and plantar pressure are critical information for footwear design and clinical assessment. The aim of this study was to investigate the relationship between plantar soft tissue hardness and plantar pressure during walking.

**Methods:**

59 healthy volunteers (27 males and 32 females, aged 20 to 82) participated in this study. The plantar surface was divided into five regions: lateral rearfoot, medial rearfoot, lateral midfoot, lateral forefoot, and medial forefoot, and the plantar tissue hardness was tested using Shore durometer in each region. Average dynamic pressures in each region were analyzed for the five regions corresponding to the hardness tests. The relationship between hardness and average dynamic pressure was analyzed in each region.

**Results:**

The average hardness of the plantar soft tissue in the above five regions is as follows: lateral rearfoot (34.49 ± 6.77), medial rearfoot (34.47 ± 6.64), lateral midfoot (27.95 ± 6.13), lateral forefoot (29.72 ± 5.47), and medial forefoot (28.58 ± 4.41). Differences of hardness were observed between age groups, and hardness of plantar soft tissues in forefoot regions increased with age (*P* < 0.05). A negative relationship was found between plantar soft tissue hardness and pressure reduction at lateral rearfoot, medial rearfoot, and lateral midfoot (*P* < 0.05).

**Conclusion:**

The hardness of plantar soft tissues changes with age in healthy individuals, and there is a trend of increasing hardness of the plantar soft tissue with age. The plantar soft tissue hardness increases with plantar pressure.

## 1. Introduction

The plantar soft tissues play a key role in absorbing shock and attenuating excessive stresses during walking, particularly in the heel-strike and push-off phases during gait [1, 2]. However, the cushioning capacity of these tissues may be impaired because of aging [3–5], diabetes [6–9], and related foot structural deformities. These problems may eventually lead to increased plantar pressures, which may contribute to foot pain, tissue damage, and high risk of fall in elderly [10].

Numerous studies have focused on measuring plantar pressure and the factors attributed to high plantar pressure, such as foot posture (normal, planus, and cavus) [11, 12], overweight due to obesity [13], gender, age, and walking speed [14]. Abnormally high plantar pressure could be mitigated by offloading or load-redistributing strategies with various therapeutic insole and/or footwear [15, 16]. Measuring the plantar pressure distribution during walking is a standard practice for designing orthoses and shoe insoles.

A therapeutic insole must be able to alter harmful plantar load distributions to relieve pain or local symptoms in the diseased foot. However, the primary goal of most existing therapeutic insole designs is geometrical fitting of the shape of plantar surface. An improved loading transfer is also dependent on how well the material characteristics of the insole match with the intrinsic mechanical property of plantar soft tissues. Thus, the knowledge of the material properties of plantar soft tissues is critical for footwear design and clinical assessment that may lead to improved treatment options, such as a suitable insole design that that are impedance matching with the plantar soft tissue [17, 18]. Plantar soft tissues are a composite material composed of fatty and various connective tissues. To quantify the material properties of regional plantar soft tissues, various researchers conducted in vivo tests with a tissue ultrasound palpation system [5, 6] and in vitro tests using material compression testing machines [17, 19]. These tests revealed that plantar soft tissues have region-specific material properties at the heel, metatarsal heads, and big toe. Previous studies reported that the stiffness of plantar soft tissues considerably increases with age [3–5]. A study examined the effects of gender, body mass (BM), and BM index (BMI) on the stiffness of plantar soft tissues by using an in vivo tissue indenter. The authors indicated that BM and BMI are weakly associated with plantar tissue stiffness, and gender difference does not affect stiffness among the elderly [20].

While many have focused on plantar pressure or regional plantar soft tissue properties to design more effective orthotic insoles, and regional differences are examined, little attention has been given to investigate the relationship between plantar soft tissue hardness and plantar pressure in healthy population. We speculate that the region-specific material properties of plantar soft tissues may be attributed to tissue adaptation to physical stress (plantar pressure) as explained by physical stress theory [21]. Studies have revealed that plantar pressure is associated with the formation of plantar calluses and addressed plantar calluses that develop in regions of increased pressure [22, 23]. However, the relationship between the hardness of plantar soft tissues and plantar pressure in healthy populations (i.e., without calluses) is still unknown.

The testing methods, such as the use of a material compression testing machine or a tissue ultrasound palpation system, adopted in previous studies are complicated to implement for footwear design and clinical assessment. Moreover, the parameters tested, such as elastic modulus, are difficult to match with Shore hardness, a scale commonly used in footwear design to evaluate the hardness of insole materials.

In the present study, we used a Shore durometer to quantify the hardness of plantar soft tissues. This testing method is easy to implement, and the testing results can be readily compared with the provided material properties of footwear to design insoles that match with the impedance of plantar soft tissues. We evaluated the probable influence of gender, aging, and BMI on hardness. Our main objective was to determine the intrinsic relationship between plantar soft tissue hardness and plantar pressure in healthy people. We hypothesize that the location of hard soft tissues corresponds with areas of high plantar pressures.

## 2. Materials and Methods

### 2.1. Participants

A total of 65 participants (aged 19 to 82) volunteered in this study. Volunteers were excluded if they had the following conditions: (1) plantar corns and calluses, (2) hallux valgus and lesser toe deformities, (3) diabetes, and (4) any abnormality in the lower extremity that may affect gait. Previous studies have demonstrated that these diseases or deformities affect plantar soft tissue hardness or plantar pressure [7, 23, 24].

### 2.2. Measurement of Hardness of Regional Plantar Soft Tissues

Hardness tester instruments were used in previous studies to measure the hardness of soft tissues [25, 26]. We used a similar Shore durometer (GS-754G, Type OO, TECKOCK, Japan) to measure the hardness of plantar soft tissues. A Shore OO durometer was designed to test the hardness of soft materials that are easy to distort, such as a sponge rubber and plastic foams (their hardness is close to that of plantar soft tissues). The radius of the indenter was 1.19 mm, which did not cause discomfort to the participants during the indentation test. The durometer reads the Shore values from 0 to 100, and it was inspected periodically for precision before each trial.

All of the hardness testing was conducted among 9:00-11:00 am. During the test, each subject was asked to rest for 10 min in nonweight bearing condition. Then, the participants were asked to lie in a supine position with their feet in neutral position during the test. The Shore durometer was pressed to the plantar surface of the foot while keeping its bottom surface in parallel with the plantar surface, as shown in Figure 1. The number on the dial plate represented the Shore hardness of the plantar soft tissue, and the durometer read the hardness in degree Shore OO. Softer tissue has lower Shore value, and harder tissue has higher Shore value. The plantar surface was divided into five regions: lateral rearfoot, medial rearfoot, lateral midfoot, lateral forefoot, and medial forefoot. Each region was measured thrice. At lateral forefoot, the 3^th^,4^th^, and 5^th^ metatarsal head areas were measured; at medial forefoot, the 1^st^ and 2^nd^ metatarsal head areas and big toe were measured.

### 2.3. Measurement of Plantar Pressure

Plantar pressures were measured while walking barefoot on a level ground by using a plantar pressure system (Diasu Dual Platform 2D, Sa.Ni Corporate s.r.l., Rome/Italy). The system has multiple sensor arrays with a special resolution of 4 sensors/cm^2^. A two-step initiation protocol was implemented to collect plantar pressure data, and this protocol has a good retest reliability and can minimize the influence of walking speed on plantar pressure variabilities [27, 28]. All participants were situated two steps away from the platform and asked to walk at their comfortable pace. They were told to walk straight and not to look at the platform during the trials. Milletrix Software (version 49) was used to analyze the dynamic plantar pressures measured by the platform (Figure 2). The dynamic maximum peak pressure for each foot and the average pressures were analyzed for the five regions corresponding to the hardness tests (namely, lateral rearfoot, medial rearfoot, lateral midfoot, lateral forefoot, and medial forefoot). Pressure reduction in the five foot regions was assessed relative to the dynamic maximum peak pressure under each foot as follows:

(1) $$\begin{array}{c} P.\text{reduction}=\frac{P.\mathrm{Max}-\text{Avg}.P}{P.\mathrm{Max}}\times 100\%, \end{array}$$

where *P*.reduction is the pressure reduction in each region, Avg.*P* is the average pressure in each region, and *P*.Max is the dynamic maximum peak pressure under each foot.

### 2.4. Statistical Analysis

The data of bilateral feet were collected, and statistical analyses were performed using SPSS version 20.0 (SPSS Inc., IBM Armonk, NY, USA). The influences of the participants' general characteristics on plantar soft tissue hardness were analyzed using one-way ANOVA. When significant findings were obtained, Bonferroni post hoc analyses were performed to examine group differences. The correlation between plantar soft tissue hardness and pressure reduction was analyzed using Pearson correlation coefficients. The level of significance was set at *P* < 0.05.

## 3. Results

Six volunteers were excluded, whereas 59 volunteers (32 females and 27 males) were included in this study. Their general characteristics are presented in Table 1. The mean hardness (Shore OO value) of plantar soft tissues and the average dynamic plantar pressures in the five foot regions are presented in Table 2, respectively.

### 3.1. Effects of Age, Gender, and BMI on the Hardness of Regional Plantar Soft Tissues

The effects of age, gender, and BMI on the hardness of plantar soft tissues were analyzed independently using one-way ANOVA. Differences were observed between age groups in forefoot regions (lateral forefoot and medial forefoot) (*P* < 0.05). The results showed that the Shore hardness of plantar soft tissues in forefoot regions increased with age (*P* < 0.05) (Table 3, Figure 3). The plantar soft tissues at rearfoot and midfoot regions tended to be harder with increasing age, from the softest for the group aged 20–39 years to the hardest for the over 60 years age group (Figure 3). However, this difference did not reach the level of significance (*P* > 0.05, Table 3).

Females exhibited lower plantar tissue hardness in the rearfoot and midfoot regions but harder tissues in the forefoot regions than the males. However, no statistical differences were observed (Table 4, *P* > 0.05). BMI was found to have no significant association with plantar soft tissue hardness (*P* > 0.05).

### 3.2. Relationship between Plantar Tissue Hardness and Plantar Pressure

Pressure reduction in the five foot regions were calculated from the dynamic maximum peak pressure under each foot and the average pressure in each region, and the average pressure reduction in the five regions is presented in Table 5. The Pearson correlation coefficients for comparison between plantar soft tissue hardness and pressure reduction in the five foot regions are presented in Table 6. A negative relationship was observed between plantar soft tissue hardness and pressure reduction at the lateral rearfoot (*P* = 0.001), medial rearfoot (*P* = 0.009), and lateral midfoot (*P* = 0.009). A low correlation coefficient was noted at the lateral and medial forefoot regions (*P* > 0.05).

## 4. Discussion

The first aim of this study was to evaluate the influence of aging, gender, and BMI on the hardness of plantar soft tissues by using a Shore durometer. We compared the average hardness of plantar soft tissues among the age groups. Results confirmed that individuals in different age groups may have different plantar soft tissue hardness. Particularly, in the forefoot regions, there was a significant difference in plantar soft tissue hardness between different age groups (*P* < 0.05), it revealed that the hardness of plantar soft tissues in forefoot regions increased with age. While no statistical differences were observed between the hardness of plantar soft tissues at rearfoot and midfoot regions (*P* > 0.05, Table 3), the plantar soft tissues also tended to be harder with increasing age, and the group aged 20–39 years have softest plantar soft tissue, as hardest for the over 60 years age group (Figure 3). Similarly, correlations between age and hardness of the plantar soft tissues were reported in the literature [3, 5]. Kwan et al. [5] examined the plantar soft tissue of sixty healthy volunteers (aged from 41 to 83 years) and measured the stiffness of the plantar soft tissues under the big toe, first metatarsal head, third metatarsal head, fifth metatarsal head, and heel. The authors compared the plantar soft tissue hardness between four age groups and found strong positive correlations between age and stiffness of the plantar soft tissues in above five foot regions (*P* < 0.01). At the forefoot regions, our results agreed with the previous study, but differences at rearfoot and midfoot regions between age groups were insignificant (*P* > 0.05). In the present study, the device we used to measure plantar soft tissue hardness was different from that of the previous study, which employed an ultrasound palpation system [5]. These factors may explain the discrepancy in the results. In the present study, the results revealed that the hardness of plantar soft tissues appear to change with age in healthy individuals, and there is a trend of increasing hardness of the plantar soft tissue with age, the results are generally consistent with those of previous studies.

For different gender groups, the present study found no significant association between gender and plantar soft tissue hardness (Table 4, *P* > 0.05). These results are similar to the findings of previous studies [20, 29]. A study reported significant differences in the hardness of plantar soft tissues in the heel region between males and females, but the researchers analyzed individuals over 71 years old only [5]. By contrast, we found that there were general trends that females had lower plantar tissue hardness in rearfoot and midfoot regions than males among all age groups, as shown in Figure 4. In addition, the females had harder plantar tissue at the forefoot than the males, a result that was not reported in previous studies. This trend may be due to the use of high-heeled shoes by females that kept their metatarsophalangeal (MTP) joints extended for long durations and which may have changed the material properties of their soft tissues under the forefoot [30].

No significant effects of BMI on plantar soft tissue hardness were observed. This result agrees with that of previous studies [4, 20].

The second aim of this study was to determine a possible relationship between the hardness of regional plantar tissues and the average plantar pressure patterns measured during walking. Results showed that plantar soft tissues had region-specific material properties and plantar pressures, as shown in Figure 5. The results agree with those of previous studies [17, 31]. Goffar et al. [31] measured the plantar pressure for 115 participants using an in-shoe pressure measurement system; their results demonstrated that plantar soft tissues had borne region-specific plantar pressures. Ledoux and Blevins [17] investigated the material properties of the plantar soft tissue from six different plantar locations in vitro, analyzed tissue modulus, energy loss, and their results showed that plantar soft tissues had region-specific material properties. In the present study, we compared the hardness of regional plantar soft tissues with pressure reduction in five foot regions. Results revealed a negative relationship between plantar tissue hardness and average pressure reduction at the lateral rearfoot, medial rearfoot, and lateral midfoot (Table 6, *P* < 0.01). In other words, higher average plantar pressures were observed for regions where plantar soft tissue were harder for the above three regions. These findings suggest that the plantar pressure at the rearfoot and midfoot can be predicted through the measurement of plantar tissue hardness. Interestingly, at the forefoot regions, the results indicated no significant correlation exists between plantar tissue hardness and plantar pressure. It may be explained by the fact that at the forefoot, MTP joint motion may have an impact on regional forefoot plantar tissue hardness, as the MTP joints dorsiflexed the soft tissue under MTP joints become “tightened,” and previous studies have reported such observation [32–34]. This also means that soft tissue hardness under the MTP joints will subject to change with the MTP joint angle. In the present study, the hardness of plantar soft tissues was tested in a neutral position. This set up may not truly reflect the hardness of plantar soft tissues at the forefoot during push-off phase in walking.

Although a number of researchers have examined the material properties of regional plantar soft tissues [6, 17–19, 33], their findings are not widely applicable to designing orthopedic insoles compared with those of studies that assessed plantar pressure [15, 16], because the methods adopted to test the properties of plantar soft tissues are difficult to implement during footwear design and clinical assessment. In the present study, the testing method was similar to that for testing the hardness of footwear materials and could be used for designing orthopedic insoles which are impedance matched with plantar soft tissues. Our findings provide the basis for designing effective orthopedic insoles that consider the association between plantar pressure distribution and plantar soft tissue properties and promote a combination of the plantar pressure and regional plantar soft tissue property.

A limitation of this study is the manual measurement of tissue hardness. Such a method may be easily affected by anthropic factors. Moreover, we did not measure the hardness in the forefoot regions at different MTP joint angles. The different angles may correspond to dynamic plantar pressures at the forefoot. We recognize that the hardness of plantar soft tissues as tested in a neutral position may not fully represent the hardness of the forefoot soft tissues during walking.

## 5. Conclusion

This study confirmed the influence of aging on the hardness of plantar soft tissues among healthy individuals. The hardness of plantar soft tissues appears to change with age in healthy individuals, and there is a trend of increasing hardness of the plantar soft tissue with age. We have provided preliminary data demonstrating a positive relationship between the hardness of plantar soft tissues and the plantar pressure distribution at the rearfoot and midfoot. These findings are important to understand the effects of physical stress (plantar pressure) on the hardness of regional plantar soft tissues.

## Figures and Tables

**Figure 1:** Measurement of plantar soft tissue hardness by using the Shore (OO) durometer. The results were averaged for the effective hardness based on the above five regions.

**Figure 2:** Schematic illustration of foot pressure areas determined by the plantar pressure testing system. The five regions corresponding to the hardness tests were analyzed.

**Figure 3:** Average plantar soft tissue hardness in the five regions among age groups (RF: rearfoot; MF: midfoot; FF: forefoot).

**Figure 4:** Analysis average plantar soft tissue hardness in the five regions between gender groups (RF: rearfoot; MF: midfoot; FF: forefoot).

**Figure 5:** Average hardness (a) and average dynamic pressure (a) in the five regions tested.

**Table 1:** General characteristics of participants (mean ± SD) (*n* = 59; BMI: body mass index; F: female; M: male).

Gender	Age (y)	Height (m)	Weight (kg)	BMI (kg/m^2^)
F (32), M (27)	43.90 ± 17.58	1.67 ± 0.08	64.01 ± 11.14	22.84 ± 3.25

**Table 2:** Plantar soft tissue hardness and dynamic plantar pressure (mean ± SD) (*n* = 59, 118 feet. RF: rearfoot; MF: midfoot; FF: forefoot).

Foot regions	Lateral RF	Medial RF	Lateral MF	Lateral FF	Medial FF
Hardness (Shore OO)	34.49 ± 6.77	34.47 ± 6.64	27.95 ± 6.13	29.72 ± 5.47	28.58 ± 4.41
Dynamic P (g/cm^2^)	586.40 ± 103.48	568.45 ± 107.70	546.56 ± 137.16	543.40 ± 115.17	572.04 ± 111.35

**Table 3:** Comparison of plantar soft tissues hardness (mean ± SD) between age groups.

	Foot regions	Age groups			F	P
		20-39 (*n* = 29)	40-59 (*n* = 15)	≥60 (*n* = 15)		
Right foot	Lateral RF	33.26 ± 6.90	34.17 ± 4.41	36.40 ± 6.82	1.053	0.356
	Medial RF	33.31 ± 6.66	34.17 ± 3.81	37.03 ± 8.86	1.529	0.226
	Lateral MF	26.36 ± 6.47	28.27 ± 4.18	29.91 ± 6.67	1.789	0.176
	Lateral FF	26.93 ± 4.50	28.43 ± 4.81	31.60 ± 5.49	6.610	0.003
	Medial FF	27.25 ± 4.17	28.21 ± 2.59	31.44 ± 4.97	5.295	0.008

Left foot	Lateral RF	32.79 ± 5.79	34.67 ± 7.33	35.11 ± 6.03	1.096	0.359
	Medial RF	32.20 ± 6.32	33.86 ± 5.00	36.83 ± 8.25	0.947	0.424
	Lateral MF	26.66 ± 5.83	29.20 ± 5.07	29.88 ± 7.67	1.231	0.307
	Lateral FF	28.15 ± 4.02	30.53 ± 5.21	33.54 ± 7.36	3.797	0.015
	Medial FF	27.08 ± 4.09	28.25 ± 3.46	31.84 ± 4.87	4.380	0.008

**Table 4:** Comparison of plantar soft tissues hardness (mean ± SD) between gender differences.

Left foot	Age	Foot regions				
		Lateral RF	Medial RF	Lateral MF	Lateral FF	Medial FF
Male	39.37 ± 17.38	35.56 ± 7.32	35.3 ± 6.8	29.00 ± 5.91	28.82 ± 4.51	28.41 ± 4.42
Female	47.72 ± 17.23	33.97 ± 6.3	33.75 ± 6.31	27.45 ± 6.41	31.31 ± 6.31	28.75 ± 4.61
*P* value		0.327	0.313	0.341	0.092	0.775
Right foot						
Male	39.37 ± 17.38	35.15 ± 7.45	35.33 ± 7.19	29.00 ± 6.4	28.00 ± 4.82	28.25 ± 4.51
Female	47.72 ± 17.23	33.56 ± 6.27	33.75 ± 6.48	26.69 ± 5.76	30.32 ± 5.51	28.82 ± 4.3
*P* value		0.367	0.365	0.150	0.094	0.618

**Table 5:** Average pressure reduction (mean ± SD) in the five regions.

Foot regions	Lateral RF	Medial RF	Lateral MF	Lateral FF	Medial FF
Pressure reduction (%)	54.70 ± 10.99	52.92 ± 10.83	51.14 ± 13.83	50.39 ± 9.94	53.17 ± 10.36

**Table 6:** Pearson correlation coefficient analysis of comparing plantar soft tissue hardness with pressure reduction.

Foot regions	Lateral RF	Medial RF	Lateral MF	Lateral FF	Medial FF
Pressure reduction (%)	54.70 ± 10.99	52.92 ± 10.83	51.14 ± 13.83	50.39 ± 9.94	53.17 ± 10.36
Pearson correlation	-0.309	-0.240	-0.251	-0.087	-0.142
*P*	0.001	0.009	0.006	0.347	0.126

## Data Availability

The data are made available through the corresponding authors' emails.
